The article "MiR-186-5p Downregulates NAMPT and Functions as a Potential Therapeutic Target for Sepsis-Induced Coagulation Disorders" was retracted in 2022. Reason: concerns about the peer review.

# MiR-186-5p Downregulates NAMPT and Functions as a Potential Therapeutic Target for Sepsis-Induced Coagulation Disorders

**DOI:** 10.1155/2022/1714041

**Published:** 2022-06-02

**Authors:** Hao Shen, Keliang Xie, Min Peng, Xiaoye Wang

**Affiliations:** Department of Intensive Care Unit, Tianjin Medical University General Hospital, Tianjin 300052, China

## Abstract

**Purpose:**

Present study is aimed to explore the role of miR-186-5p in sepsis-induced coagulation disorders and molecular mechanisms.

**Methods:**

Thirty-four sepsis patients and 34 respiratory infection/pneumonia patients were selected in the present study. Polymicrobial sepsis model was created by cecal ligation and puncture (CLP). The mRNA expression was detected by qRT-PCR. Western blot was utilized to measure protein expression. Thromborel S Reagent was applied to measure the prothrombin time (PT). Platelet count of blood was measured via LH 780. ELISA kits were utilized to evaluate the fibrinogen and PAI-1 concentration.

**Results:**

MiR-186-5p expression was lower and nicotinamide phosphoribosyltransferase (NAMPT) mRNA expression was higher in sepsis patients in contrast to control group. Coagulation time was markedly prolonged and platelet count was markedly decreased in CLP mice. In addition, fibrinogen concentration was obviously lower and PAI-1 concentration was obviously higher in CLP mice. MiR-186-5p mimic obviously decreased coagulation time and PAI-1 concentration, while raised platelet count and fibrinogen concentration. Targetscan predicted miR-186-5p might directly regulates NAMPT, and luciferase reporter assay verified this prediction. In addition, miR-186-5p mimic obviously inhibited the mRNA expression of NAMPT. Knockdown of NAMPT improved coagulation dysfunction in sepsis. Overexpression of NAMPT reversed the improvement effect of miR-186-5p on coagulation dysfunction. MiR-186-5p mimic markedly inhibited NF-*κ*B pathway.

**Conclusion:**

MiR-186-5p inhibited sepsis-induced coagulation disorders via targeting NAMPT and inactivating NF-*κ*B pathway.

## 1. Introduction

Sepsis is a multiorgan dysfunction caused by the maladjusted response of the host to infection, which seriously threatens human health [1]. Sepsis is a common complication of severe trauma, burn, shock, infection, and so on [2]. Systemic inflammatory reaction can affect many organs such as kidney, liver, lung, and so on. With the continuous improvement of medical level, the incidence and mortality of sepsis have been greatly reduced. However, sepsis has caused great pressure and harm to medical treatment and patients all over the world. About 49 million people worldwide are infected with sepsis every year, and about 5 million people died of sepsis every year [3]. Multiple organ failure caused by sepsis is an important reason for the high mortality of sepsis. Multiple organ failure is mainly due to the oxidative stress response induced by a large number of inflammatory factors produced by sepsis, resulting in endothelial cell injury and microvascular thrombosis [4]. Extensive microvascular thrombosis leads to tissue ischemia and cell hypoxia, resulting in organ injury and dysfunction, and even organ failure. Thrombosis is closely related to platelets and coagulation mechanism. Thrombocytopenia and abnormal coagulation function are common pathological processes in the progression of sepsis [2]. In the process of sepsis, strong inflammatory reaction activates proinflammatory cells, various cytokines, and chemokines, resulting in the activation of coagulation system. Activation of the coagulation system leads to thrombosis and disseminated intravascular coagulation. This study intended to explore the role of miR-186-5p in sepsis-induced coagulation dysfunction and related mechanism.

The article "MiR-186-5p Downregulates NAMPT and Functions as a Potential Therapeutic Target for Sepsis-Induced Coagulation Disorders" was retracted in 2022. Reason: concerns about the peer review.

MicroRNA (miRNA) is a small molecule non-coding regulatory RNA, which was found in Nematoda in 1993 [5]. miRNA is composed of about 20–23 endogenous noncoding nucleotides, which can bind to miRNA to inhibit its translation or promote its degradation. miRNA is involved in regulating various physiological processes of the body, such as cell metabolism, proliferation and differentiation, growth and apoptosis [6]. miRNA plays an important regulatory role in the occurrence and development of many diseases. The changes of miRNA can also affect the occurrence and development of diseases and individual sensitivity to drug therapy [7]. miRNA provides new ideas for us to deeply understand the occurrence and development of various diseases at the molecular level.

Many studies have shown that miRNAs were involved in sepsis-induced organ failure and coagulation disorder. For instance, miR-23a improved sepsis lung injury through PI3K/Akt/*p*53 pathway [8]. MiR-21 and miR-181b targeted NFI-A to enhance resistance to sepsis infection [9]. Overexpression of miR-21 had a protective effect on sepsis-induced renal cell apoptosis through PTEN/PI3K/Akt signaling pathway [10]. However, the role of miR-186-5p in sepsis is still unclear.

Hence, the purpose of this study was to explore whether miR-186-5p could attenuate coagulation disorders induced by sepsis.

## 2. Materials and Method

### 2.1. Human Sample

The blood samples from 34 sepsis patients and 34 respiratory infection/pneumonia patients (control group) were acquired in the hospital from September 2018 to April 2020.

### 2.2. Animals

Male mices of 8-16-week were chosen for further experiment. C57BL/6 were obtained from the ZHBY biotech Co. Ltd. (Nanchang, China) and previously crossed into the C57BL/6 strain. All mice were fed pathogen-free diet. Mice were housed under pathogen -ree and temperature-controlled conditions with 12-hour light/dark cycles.

The article "MiR-186-5p Downregulates NAMPT and Functions as a Potential Therapeutic Target for Sepsis-Induced Coagulation Disorders" was retracted in 2022. Reason: concerns about the peer review.

### 2.3. Cecal Ligation and Puncture Model of Polymicrobial Sepsis

Polymicrobial sepsis was created by cecal ligation and puncture (CLP) as previously described [11,12]. Each mice was injected with miR-186-5p mimic, si-nicotinamide phosphoribosyltransferase (si-NAMPT), and corresponding negative control (Genechem, China).

### 2.4. Blood Collection and Examination

Whole blood was collected via cardiac puncture under general anesthesia and transferred to 1 mL capillary blood collection tubes containing 3.2% sodium citrate (Absin, China). The prothrombin time (PT) was measured via Thromborel S Reagent (Siemens, Germany). Platelet count of blood was measured via LH 780 (Coulter LH, USA). ELISA kits (Corning, USA) were applied to detect the fibrinogen and PAI-1 concentration.

2.5 RNA Isolation and Quantitative Real-Time PCR Analysis Total RNA was extracted from cells via the RNA extraction kit (Beyotime, China). After measuring the purity and concentration of RNA by a microquantitative nucleic acid meter, it was transferred to cDNA according to the reverse transcription kit (Absin, China). RT-qPCR amplification was then performed using cDNA as the template. Relative expression of miR-186-5p and NAMPT mRNA was calculated by the 2^-△△Ct^ method.

### 2.5. Western Blot

RIPA reagent was applied to extract the total protein in cells (Absin, China), and BCA protein kit (Corning, USA) was applied to measure the protein content. After protein denaturation, 10% SDS-PAGE electrophoresis was performed. After protein denaturation, 10% SDS-PAGE electrophoresis was performed. After electrophoresis, the separated protein was transferred to PVDF membrane and sealed with 5% skimmed milk powder for 1.5 h. First antibody (1 : 1000, Abcam, U K) was added and incubated overnight at 4°C. Goat antirabbit secondary antibody (1 : 2000, Abcam, U K) was added and incubated at 37°C for 2h.

### 2.6. Luciferase Reporter Assay

The HEK 293T cells (Beyotime, China) were used for luciferase reporter assay. The WT and MUT sequences of NAMPT were synthesized by Tingske Biotechnology Co., Ltd. We inserted the wild-type (WT) or mutant (MUT) of miR-186-5p binding site in 3′UTR into the pGL3 vector (Promega, USA). The HEK 293T cells were co-transfected with NAMPT-WT or NAMPT-MUT and miR-186-5p by Lipofectamine. The luciferase activity was measured after transfection for 48 h using Dual-Luciferase Reporter Assay System.

The article "MiR-186-5p Downregulates NAMPT and Functions as a Potential Therapeutic Target for Sepsis-Induced Coagulation Disorders" was retracted in 2022. Reason: concerns about the peer review.

### 2.7. Statistical Analysis

Data was analysed via SPSS.25. Differences of groups were compared using one-way analysis of variance (ANOVA) and *t*-test. *P* values less than 0.05 were considered statistically significant.

## 3. Results

### 3.1. The Expression of miR-186-5p Decreased in Sepsis Patients

In contrast to the control group, miR-186-5p was lower expressed in sepsis patients, as shown in Figure 1(a). In contrast to the control group, NAMPT mRNA expression was higher expressed in sepsis patients, as shown in Figure 1(b).

### 3.2. MiR-186-5p Improved Coagulation Dysfunction in Sepsis

CLP mice showed the characteristics of prolonged coagulation time and decreased platelet count (Figure 2(b)). In addition, CLP mice had obviously lower fibrinogen concentration and higher PAI-1 concentration (Figures 2(c) and 2(d)). However, miR-186-5p obviously decreased coagulation time and raised platelet count (Figures 2(a) and 2(b)). MiR-186-5p obviously raised fibrinogen concentration and decreased PAI-1 concentration (Figure 2(c) and 2(d)).

### 3.3. MiR-186-5p Directly Regulated the Expression of NAMPT

Next, we used targetscan and luciferase reporter assay to analyze the relationship between miR-186-5p and NAMPT. NAMPT was predicted to be regulated via miR-186-5p (Figure 33(a)). MiR-186-5p obviously decreased luciferase activity of NAMPT-WT while miR-186-5p did not change luciferase activity of NAMPT-MUT (Figure 3(b)). In addition, miR-186-5p mimic obviously raised the expression of miR-186-5p (Figure 3(c)) and inhibited the mRNA expression of NAMPT (Figure 3(d)).

### 3.4. Knockdown of NAMPT Improved Coagulation Dysfunction in Sepsis

Knockdown of NAMPT obviously decreased coagulation time and raised platelet count (Figures 4(a) and 4(b)). Knockdown of NAMPT obviously raised fibrinogen concentration and decreased PAI-1 concentration (Figures 4(c) and 4(d)).

### 3.5. Overexpression of NAMPT Reversed the Improvement Effect of miR-186-5p on Coagulation Dysfunction

Overexpression of NAMPT obviously increased coagulation time and raised platelet count (Figures 5(a) and 5(b)). Overexpression of NAMPT obviously raised fibrinogen concentration and decreased PAI-1 concentration (Figures 5(c) and 5(d).

### 3.6. MiR-186-5p Inhibited NF-Κb Pathway

In order to study whether miR-186-5p affects NF-*κ*B signal pathway, we detected the protein expression by Western blot assay. LPS obviously activated the NF-*κ*B signal pathway, while miR-186-5p mimic inhibited it (Figure 6).

## 4. Discussion

Sepsis is a complex multisystem disease, which is related to environmental, genetic, and metabolic factors [2]. It is characterized by the maladjusted response of the host to infection. More than 80% of patients with sepsis have different degrees of coagulation disorders, and the mortality of these patients is much higher [2]. Sepsis can lead to coagulation dysfunction, including decreased platelet, prolonged coagulation time, and increased risk of thrombosis. In severe cases, fulminant disseminated intravascular coagulation (DIC) characterized by spontaneous diffuse microvascular thrombosis and multisite bleeding can occur. The continuous reduction of platelets and coagulation factors increases the risk of intravascular coagulation disorders and bleeding [4]. In sepsis, infection can lead to inflammatory response and systemic inflammatory response syndrome. There is a large amount of evidence that there is an important association between inflammation and coagulation dysfunction. Inflammation and coagulation dysfunction may play an important role in the pathological process of organ failure in patients with sepsis [13]. Inflammation can not only lead to the activation and development of coagulation dysfunction but also affect the development of inflammation [2].

The article "MiR-186-5p Downregulates NAMPT and Functions as a Potential Therapeutic Target for Sepsis-Induced Coagulation Disorders" was retracted in 2022. Reason: concerns about the peer review.

In this study, the CLP mice model was established firstly. CLP mice showed the characteristics of prolonged coagulation time and decreased platelet count. In addition, CLP mice had obviously lower fibrinogen concentration and higher PAI-1 concentration. The disorder of coagulation function in sepsis will lead to the loss of coagulation factors in patients with sepsis. Coagulation dysfunction in sepsis can be manifested by the decrease of plasma fibrinogen level. Platelets are important regulators of inflammation and hemostasis. They are the first cells to reach the site of acute injury and interact with endothelial cells and leukocytes. In patients with severe sepsis, there is almost always a decrease in platelet count. Studies have shown that about 14% to 28% of patients in intensive care unit will have prolonged coagulation time, such as prothrombin time or activated partial thromboplastin time [14]. We found miR-186-5p obviously decreased coagulation time and PAI-1 concentration, which was lower expressed in sepsis patients, while raised platelet count and fibrinogen concentration. These results indicated miR-186-5p improved coagulation dysfunction in sepsis. Some studies have demonstrated that miRNAs are involved in coagulation disorders [15–17]. For instance, miR-19a-3p inhibited disseminated intravascular coagulation induced by sepsis through binding to TF [15]. MiR-186-5p affects tumor progression through a variety of ways, including regulating target genes to inhibit cell growth, promoting cell cycle arrest and apoptosis, preventing tumor cell invasion and metastasis, and reducing tumor angiogenesis and lymphangiogenesis [18].

The article "MiR-186-5p Downregulates NAMPT and Functions as a Potential Therapeutic Target for Sepsis-Induced Coagulation Disorders" was retracted in 2022. Reason: concerns about the peer review.

The role of miRNA is to negatively regulate the expression of a gene. Subsequently, Targetscan predicted NAMPT was regulated via miR-186-5p, and luciferase reporter assay verified this conjecture. NAMPT was higher expressed in sepsis patients. MiR-186-5p obviously decreased luciferase activity of NAMPT-WT while miR-186-5p did not change luciferase activity of NAMPT-MUT. In addition, miR-186-5p mimic obviously inhibited the mRNA expression of NAMPT. Overexpression of NAMPT reversed the improvement effect of miR-186-5p on coagulation dysfunction. These results suggested that miR-186-5p can alleviate sepsis-induced coagulation disorder by regulating NAMPT. NAMPT is the rate limiting enzyme of NAD + remedial synthesis pathway. It has a variety of important physiological functions and plays an important role in the regulation of energy metabolism [19]. NAMPT plays an important role in cell metabolism and immune regulation. At the same time, it can also induce inflammatory response as a cytokine [20, 21]. Studies have shown that NAMPT was increased in inflammatory environment, such as diabetes, inflammatory bowel disease, rheumatoid arthritis, and myocardial infarction [21, 22]. Koch et al. found that the level of NAMPT in serum can predict the mortality of patients with sepsis [23]. MiR-96-5p relieved inflammatory response by binging to NAMPT and inactivating NF-*κ*B pathway sepsis [6]. In the present study, we also found miR-186-5p inhibited NF-*κ*B pathway.

NF-*κ*B pathway is an important signal transduction pathway widely existing in mammals, which is involved in many diseases such as inflammation and tumor. NF-*κ*B is activated by inflammatory factors, and IKBa and p65 are phosphorylated to enhance their transcriptional activity. Therefore, detecting the phosphorylation of iKBa and p65 could reflect p65-*κ*B activation level. Present study found miR-186-5p mimic inactivated NF-*κ*B signal pathway via suppressing the phosphorylation of iKBa and p65. NF-*κ*B is a typical transcription factor and plays a major regulatory role in sepsis. In sepsis, masses of inflammatory factors are released, activating NF-*κ*B signaling. In conclusion, miR-186-5p targeted NAMPT to inhibit sepsis-induced coagulation disorders via inactivating NF-*κ*B pathway.

## Figures and Tables

**Figure 1:** MiR-186-5p was lower expressed in sepsis patients. (a) MiR-186-5p expression was detected via qPCR. (b) NAMPT mRNA expression was detected via qPCR. ^*∗*^(*P*) < 0.05.

**Figure 2:** MiR-186-5p improved coagulation dysfunction in sepsis. (a) Prothrombin time was measured using standard kits for a Clot 2 coagulometer. (b) Platelet counts were conducted via an automated device for animals. (c), (d). ELISA kits were utilize to measure fibrinogen levels (c). and PAI-1 (d). ^*∗*^(*P*) < 0.05.

The article "MiR-186-5p Downregulates NAMPT and Functions as a Potential Therapeutic Target for Sepsis-Induced Coagulation Disorders" was retracted in 2022. Reason: concerns about the peer review.

**Figure 3:** MiR-186-5p directly regulates NAMPT. (a) Predicted binding sites. (b) Luciferase reporter assay was conducted to confirm the relationship between miR-186-5p and NAMPT. (c) MiR-186-5p expression was detected via qPCR. (d) The mRNA expression of NAMPT was measured via qPCR. ^*∗*^(*P*) < 0.05.

**Figure 4:** Knockdown of NAMPT improved coagulation dysfunction in sepsis (a). Prothrombin time was measured using standard kits for a Clot 2 coagulometer (b). Platelet counts were conducted via an automated device for animals (c), (d). ELISA kits was utilized to measure fibrinogen levels (c). PAI-1 (d). ^*∗*^(*P*) < 0.05.

**Figure 5:** Overexpression of NAMPT reversed the improvement effect of miR-186-5p on coagulation dysfunction. (a) Prothrombin time was measured using standard kits for a Clot 2 coagulometer. (b) Platelet counts were conducted via an automated device for animals. C,D. ELISA kits was utilized to measure fibrinogen levels (c). PAI-1 (d). ^*∗*^(*P*) < 0.05.

**Figure 6:** MiR-186-5p inhibited NF-*κ*B pathway. The protein expression was detected via western blot ^*∗*^(*P*) < 0.05.

## Data Availability

The data to support the findings of this study are available on reasonable request from the corresponding author.
